The article "Genetic diversity, forensic feature, and phylogenetic analysis of Guizhou Tujia population via 19 X‐STRs" was retracted in 2024. Reasons: lack of ethics approval or compliance; missing or withdrawn patient consent; no approval from an author; concerns about the data.

# Genetic diversity, forensic feature, and phylogenetic analysis of Guizhou Tujia population via 19 X‐STRs

**DOI:** 10.1002/mgg3.1473

**Published:** 2020-09-02

**Authors:** Li Luo, Hongyan Gao, Lilan Yao, Fei Long, Hao Zhang, Lushun Zhang, Yong Liu, Jian Yu, Limei Yu, Pengyu Chen

**Affiliations:** ^1^ Key Laboratory of Cell Engineering in Guizhou Province Affiliated Hospital of Zunyi Medical University Zunyi China; ^2^ Center of Forensic Expertise Affiliated Hospital of Zunyi Medical University Zunyi Guizhou China; ^3^ Shanghai Key Laboratory of Forensic Medicine Shanghai Forensic Service Platform Academy of Forensic Science Shanghai China; ^4^ Department of Forensic Biology Evidence Zunyi City Public Security Bureau Zunyi Guizhou China; ^5^ Department of Pathology and Pathophysiology Chengdu Medical College Chengdu China

## Abstract

**Background:**

X‐chromosome short tandem repeats (X‐STRs) with unique sex‐linkage inheritance models play a complementary role in forensic science. Guizhou is a multiethnic province located in southwest China and some genetic evidence focusing on X‐STRs for various minorities was reported. However, population data of Guizhou Tujia are scarce.

**Methods:**

A total of 507 Guizhou Tujia individuals were profiled using the AGCU X‐19 STR kit. Allele frequencies and forensic parameters were calculated. Additionally, population genetic relationships between Guizhou Tujia and other 19 populations were explored.

**Results:**

A total of 257 alleles with the allele frequencies ranged from 0.0013 to 0.6098 were found. The combined power of discrimination in males and females and mean exclusion chances in all case scenarios were all greater than 0.99999. Population comparisons showed Guizhou Tujia had a homogeneity with all Han populations from different administrative regions, and other ethnic populations residing in Guizhou, while had obviously genetic heterogeneity with the Altaic family populations except Xibe.

**Conclusion:**

Nineteen X‐STRs can afford a reliable and informative database of Guizhou Tujia population for human identification and paternity testing, especially in complex biological relations. The genetic relationships of Chinese are significantly influenced by the geographic position and ethnolinguistic origin.

## Graphical abstract

19 X‐STRs can afford a reliable and informative database of Guizhou Tujia population for human identification and paternity testing, especially in complex biological relations. The genetic relationships of Chinese populations are significantly influenced by the geographic position and ethnolinguistic origin.

## 1 INTRODUCTION

Short tandem repeats (STRs), also called microsatellite DNA or simple sequence repeats (SSRs), are DNA regions with a motif consisting of 2–6 bp tandemly repeated unit (Ellegren, 2004). Recently, autosomal STRs have been widely used for human identification and paternity testing since the early 1990s (Chen, Guo, et al., 2018; Edwards, Hammond, & Caskey., 1991; Jobling & Gill, 2004), but there are some defects existing in mixed stains, deficiency paternity cases, and paternity cases involving blood‐relatives (Szibor, 2007). The X chromosomal is obtained from both parents in daughter, while the son only receives one X chromosomal from his mother (Diegoli, 2015). With this unique sex‐linkage inheritance model, X‐chromosomal STRs (X‐STRs) can supplement indispensable information in forensic daily work mentioned above (Diegoli, 2015). Nowadays, X‐STRs profile has become one of the standards for forensic genetic analysis (Diegoli et al., 2016). The AGCU X‐19 STRs kit (AGCU ScienTech Inc., Wuxi, Jiangsu, China), a multiplex PCR system that can amplify 19 X‐STRs synchronously, was designed and manufactured for forensic application (Chen, He, Zou, Wang, Jia, et al., 2018). This system adopts five‐dye fluorescent labeling technology and contains seven linkage groups (LG) named LG1, LG2, LG3, LG4, LG5, LG6, and LG7. LG1 (Hering et al., 2006) includes DXS10074, DXS10075, DXS10079, and DXS7132; LG2 (Edelmann, Hering, Kuhlisch, & Szibor, 2002) consists of DXS101 and DXS7424; LG3 (Sufian, Fatema, Hasan, & Akhteruzzaman., 2017) is made up of DXS10101, DXS10103, and HPRTB; LG4 (Samejima, Nakamura, & Minaguchi, 2011) contains DXS10134 and DXS7423; LG5 (Hundertmark et al., 2008) composes DXS10148, DXS10135, and DXS8378; LG6 (Edelmann, Hering, Augustin, Kalis, & Szibor, 2010) comprises DXS10159, DXS10162, and DXS10164; DXS6789 and DXS6809 form LG7 (Szibor et al., 2005). Yang et al. (2016) manifested that the 19 X‐STRs PCR multiplex system is reliable and robust, which can turn into an effective supplementary tool in forensic and kinship analyses. Up to now, the genetic characteristics of AGCU X‐19 STRs kit have been investigated in a great number of ethnic groups in China (Chen, Guo, et al., 2018; Chen, He, Zou, Wang, Jia, et al., 2018; Chen, He, Zou, Wang, Luo, et al., 2018; Guo et al., 2019; Han et al., 2019; He, Li, Zou, Li, et al., 2017; He, Li, Zou, Wang, et al., 2017; Liu et al., 2017; Meng et al., 2017; Xiao et al., 2020; Yang et al., 2017), but the population structures of Tujia are blank.

Tujia, one of the most ancient minorities in China, mainly live in the Wuling Mountains boarding Guizhou, Hunan, and Hubei Provinces, and Chongqing Municipality. According to the sixth national population census of the Chinese government, Tujia was the seventh largest minority in 55 Chinese minorities with a population of about 8 million people (http://www.stats.gov.cn/tjsj/pcsj/rkpc/6rp/index​ch.htm). Tujia has its own language which belongs to the Tibeto‐Burman language branch of the Sino‐Tibetan language family but no script. Based on the Chinese historical sources, Tujia people are the main descendants of the Ba people, an ancient tribe in southwest China formed and named between the Xia and the Shang Dynasty. In the early period, the Ba people took Enshi as the center and lived in western Hubei. With the power increasing, the Ba people gradually expanded to the whole Wuling mountain areas, southward to the Guizhou and Hunan province, eastward to Sichuan. After the Ba was defeated by the Qin, its posterity survived and renamed “Tu” in the 1206 A.D. With the stability of the chieftain system, the Tujia people residing in Hunan, Hubei, Sichuan, and Guizhou province integrated and gradually consolidated. Since 1956, Tujia has become an officially recognized independent ethnic group (https://en.wikip​edia.org/wiki/Tujia​‐people). Guizhou, located in southwest China, is demographically one of China's most diverse provinces with a unique geographical environment and historical mass migration. Approximately 4.1% of the Tujia people in China have settled in Guizhou, and becoming the fifth chiefly ethnic group in the province (https://en.wikip​edia.org/wiki/Guizhou).

Consequently, the purpose of this study was to obtain the genetic information of 19 X‐STRs from Guizhou (southwest China) Tujia populations using AGCU X‐19 STRs kit. With these highly polymorphic STRs’ allele frequencies data, we further evaluated the X‐chromosome forensic characteristics of AGCU X‐19 STRs kit in Guizhou Tujia populations and reconstructed the population genetic structure with previously reported populations (Chen, Guo, et al., 2018; Chen, He, Zou, Wang, Jia, et al., 2018; Chen, He, Zou, Wang, Luo, et al., 2018; Guo et al., 2019; Han et al., 2019; He, Li, Zou, Li, et al., 2017; He, Li, Zou, Wang, et al., 2017; He et al., 2018; Li, Li, et al., 2019; Li, Zeng, et al., 2019; Liu et al., 2017; Meng et al., 2017; Xiao et al., 2020; Yang et al., 2017; Zhang et al., 2016). Population distribution was presented in Figure S1.

## 2 MATERIALS AND METHODS

### 2.1 Population samples and ethical statement

A total of 507 (258 males and 249 females) unrelated healthy Tujia individuals from Guizhou province (southwest China) were collected in accordance with the informed consent principle. Participants were all indigenous without immigration and interracial marriage at least three generations. This study was approved by the Biomedical Research Ethics Committee of Zunyi Medical University (No. 2014‐1‐044).

### 2.2 DNA amplification and STR genotyping

DNA extraction of Tujia individuals was performed from the EDTA anticoagulant tube using salting‐out method (Miller, Dykes, & Polesky, 1988) and quantified by NanoDrop 2000c (Thermo Fisher Scientific). Approximately 2.0 ng/μl extracted DNA was amplified by ProFlex™ 3 × 32‐well PCR System (Applied Biosystems, Foster City, CA) using AGCU X‐19 STRs kit, which includes 19 X‐STR loci (DXS8378, DXS7423, DXSl0148, DXSl0159, DXSl0134, DXS7424, DXSl0164, DXSl0162, DXS7132, DXSl0079, DXS6789, DXSl01, DXSl0103, DXSl0101, DXS6809, HPRTB, DXSl0075, DXSl0074, DXSl0135) based on the operation instruction. A total of 10 μl of PCR reaction volume were employed, including 4 μl of reaction mix, 2 μl of X‐19 primers, 0.2 μl of Taq DNA polymerase, 1 μl of DNA template, and 2.8 μl of sdH_2_O (sterile deionized H_2_O). PCR condition consisted of predegeneration of 2 min at 95℃; 10 cycles of 30 s at 94℃, 1 min at 60℃, 1 min at 65℃, then 20 cycles of 30 s at 94℃, 1 min at 59℃, 1 min at 72℃; final extension of 30 min at 60 ℃, and hold at 4℃. The PCR products were detected and separated on an ABI 3500XL Genetic Analyzer (Applied Biosystems, Foster City, CA). GeneMapper ID v1.4 software was employed to identify and assign the alleles determined by fragment sizes. Positive control (9947A DNA sample) and negative control (sdH_2_O) ran in each PCR reaction system.

### 2.3 Data analysis

Allele frequencies of Guizhou Tujia males, females, and the pooled population of AGCU X‐19 STRs kit were separately calculated using the modified PowerStats v1.2 program (Promega, Madison, WI, USA). SPSS v26.0 (Hansen, 2005) was used to assess the allele frequencies differences between males and females using the Chi‐square test. Hardy‐Weinberg equilibrium (HWE), observed heterozygosity (Ho), and expected heterozygosity (He) only in females and linkage disequilibrium (LD) both in males and females were computed using the Arlequin v3.5 software (Excoffier & Lischer, 2010). Haplotype frequencies of seven LGs were counted directly. Polymorphism information contents (PIC), power of discrimination in males (PDm), and females (PDf), paternity exclusion chance (MEC) in the Trios (MEC_Krüger) (Krüger, Lichte, & Steffens., 1968), MEC_Kishida (Kishida, Fukuda, & Tamaki., 1997), MEC_Desmarais and Duos (MEC_Desmarais_Duos) (Desmarais, Zhong, Chakraborty, Perreault, & Busque, 1998) for 19 X‐STR loci were computed using the StatsX v2.0 (Lang, Guo, & Niu, 2019).

Locus by locus Fst and corresponding *p* values of 19 X‐STRs between 20 populations, as well as pairwise Nei's genetic distances based on 19 shared X‐STRs, were calculated by Arlequin v3.5 software (Excoffier & Lischer, 2010) and Phylip v3.695 (http://evolu​tion.genet​ics.washi​ngton.edu/phylip.html.). Neighbor joining tree (N‐J tree) and multidimensional scaling plots (MDS) were visualized by Mega v7.0 (Kumar, Stecher, & Tamura, 2016) and SPSS v26.0 program (Hansen, 2005) based on the Nei's genetic distances. Principal component analysis (PCA) was also constructed by SPSS v26.0 program (Hansen, 2005).

## 3 RESULTS

### 3.1 Allele frequencies and genetic diversities of 19 X‐STR loci

In the present research, we used the AGCU X‐19 kit to genotype the 19 X‐STRs in 507 volunteers (258 males and 249 females) residing in Guizhou province successfully. The Hardy‐Weinberg equilibrium (HWE) for the 19 X‐STR loci was tested using a Markov Chain with the dememorization steps of 100,000 and forecasted chain length of 1,000,000 testing based on the observed heterozygosity (Ho) and expected heterozygosity (He) in 249 unrelated healthy Tujia females (Table S1) (Nei & Roychoudhury, 1974). The values of Ho ranged from 0.5141 (DXS7423) to 0.8956 (DXS10148), while He values spanned from 0.5170 (DXS7423) to 0.9215 (DXS10135). No departures from the HWE were observed except DXS10074, DXS10075, DXS10079, and DXS10134. However, all of the studied loci accorded with HWE after Bonferroni correction (*p* > 0.05/19 = 0.0026), which explained that the selected sample could represent Guizhou Tujia population.

Allele frequencies of Tujia males and females are presented in Table S2. There were 214 alleles with the corresponding frequencies spanned from 0.002 to 0.6084 in the females and 221 alleles with the corresponding frequencies varied from 0.0039 to 0.6124 in the males. Among them, 33 alleles were only found in females with 36 in males. According to the results of the Chi‐square test, no obvious allele frequencies distribution differences (*p* > 0.05) in all 19 loci were detected between males and females (Table S3). Therefore, allele frequencies and forensic parameters of pooled population were calculated (Table S1). A total of 257 alleles were found with the allele frequencies ranged from 0.0013 to 0.6098. The allele numbers spanned from 7 at HPRTB and DXS8378 to 27 at DXS10148.

Forensic parameters including polymorphism information contents (PIC), power of discrimination in males (PDm) and females (PDf), paternity exclusion chance (MEC) in the Trios (MEC_Krüger, MEC_Kishida, MEC_Desmarais) and Duos (MEC_Desmarais_Duos) of 19 X‐STRs based on pool frequencies are performed in Table S1. The lowest PIC (0.4402), PDm (0.5206), and PDf (0.6897) were found at DXS7423, while the highest PIC (0.9124), PDm (0.9183), and PDf (0.9875) were found at DXS10135. The combined power of discrimination in males and females were 0.999999999999818 and 0.999999999999999999999668550415, respectively. The MEC_Krüger, MEC_Kishida, MEC_Desmarais, and MEC_Desmarais_Duos were 0.2527–0.8343, 0.4400–0.9124, 0.4402–0.9124, and 0.3022–0.8444 with the combined mean exclusion chances higher than 0.99999.

### 3.2 Linkage disequilibrium, haplotype frequencies, and genetic diversities of seven linkage groups

The linkage disequilibrium (LD) for 19 X‐STRs intercomparisons was calculated by permutation test using the EM algorithm (permutations number: 10,000; EM initial conditions: 2) of females (Table S4) and was conducted by exact test using a Markov chain (Chain length: 10,000; Dememorization: 1,000) in the males (Table S5) (Tillmar et al., 2017). Of 171 loci pairs, the value of 24 pairs were less than 0.05, but there is still remained one pair (DXS10103‐DXS10101) after Bonferroni correction (*p* > 0.05/171 = 0.0003) in the females. In the male individuals, there were significant differences in 25 pairs, but only five pairs (DXS10101‐DXS10075, DXS10103‐DXS10101, DXS10159‐DXS10162, DXS10162‐DXS10164, DXS10162‐DXS7423) still deviated from LD after Bonferroni correction (*p* > 0.05/171 = 0.0003).

19 X‐STRs can be clustered into seven linkage groups (LG): LG1 (Hering et al., 2006) (DXS10074‐DXS10075‐DXS10079‐DXS7132); LG2 (Edelmann et al., 2002) (DXS101‐DXS7424); LG3 (Sufian et al., 2017) (DXS10101‐DXS10103‐HPRTB); LG4 (Samejima et al., 2011) (DXS10134‐DXS7423); LG5 (Hundertmark et al., 2008) (DXS10148‐DXS10135‐DXS8378); LG6 (Edelmann et al., 2010) (DXS10159‐DXS10162‐DXS10164); LG7 (Szibor et al., 2005) (DXS6789‐DXS6809). Haplotypes containing seven linkage groups and corresponding haplotype frequencies of males were obtained (Table S6). For these seven linkage groups (LG1–7), the number of different haplotypes in Guizhou Tujia males were 188, 51, 122, 47, 187, 103, 53 respectively, in which 139 in LG1, 21 in LG2, 74 in LG3, 23 in LG4, 138 in LG5, 55 in LG6, 17 in LG7 were unique. The most common haplotypes were 16‐17‐19‐15 (5, 0.0194) in LG1, 24‐16 (32, 0.1240) in LG2, 31‐16‐13 (22, 0.0853) in LG3, 37‐15 (34, 0.1318) in LG4, 18‐24.1‐10 (5, 0.0194) in LG5, 24‐18‐10 (19, 0.0736) in LG6, and 16‐33 (20, 0.0775) in LG7. Forensic parameters of LG1–7 were presented (Table S7). The value of haplotype diversity (HD) ranged from 0.9398 (LG4) to 0.9970 (LG1). PIC spanned from 0.9427 (LG4) to 0.9931 (LG1). PDm and PDf varied from 0.9362 to 0.9931 and 0.9925 to 0.9999 with the combined power of discrimination equal to 0.999999999996714 and 0.99999999999999999999016846604, respectively. The value of MEC_Krüger, MEC_Kishida, MEC_Desmarais, and MEC_Desmarais_Duos were 0.8730–0.9910, 0.9334–0.9979, 0.9327–0.9931, 0.8783–0.9863 with the combined mean exclusion chances higher than 0.99999.

### 3.3 Population genetic differentiation among Guizhou Tujia and other 19 populations

To better understand the homogeneity and heterozygosity between Guizhou Tujia population and other Chinese populations, genetic comparisons with 19 Chinese populations belonging to seven languages families (Sinitic (Chen, He, Zou, Wang, Jia, et al., 2018; He, Li, Zou, Wang, et al., 2017; Li, Zeng, et al., 2019; Yang et al., 2017; Zhang et al., 2016), Hmong‐Mien (Han et al., 2019), Tai‐Kadai (Chen, Han, et al., 2018; Guo et al., 2019; Xiao et al., 2020), Tibeto‐Burman (He, Li, Zou, Li, et al., 2017; He et al., 2018; Yang et al., 2017), Turkic (Li, Zeng, et al., 2019; Li, Zeng, et al., 2019; Liu et al., 2017), Mogolian (Chen, Guo, et al., 2018), and Tungusic (Meng et al., 2017)) from 10 provinces were carried out based on 19 X‐STRs from published literature using locus by locus Fst, Nei's genetic distance, N‐J tree, multidimensional scaling plots (MDS), and principal component analysis (PCA) (Table S8). The reference populations contained six Sinitic‐speaking populations (Xinjiang Han, Ningxia Hui, Shaanxi Han, Sichuan Han, Guizhou Han, and Southern China Han: Guangdong, Jiangxi, Hunan, and Guangxi provinces), four Tai‐Kadai‐speaking populations (Guizhou Gelao, Guizhou Sui, Guangxi Zhuang, and Guangxi Mulao), three Tibeto‐Burman‐speaking populations (Tibet Tibetan, Sichuan Tibetan, and Sichuan Yi), one Hmong‐Mien‐speaking population (Guizhou Miao), three Turkic‐speaking populations (Xinjiang Uyghur, Xinjiang Kyrgyz, Xinjiang Kazakh), one Mogolian‐speaking population (Xinjiang Mogolian), and one Tungusic‐speaking population (Xinjiang Xibe).

Locus by locus Fst and corresponding *p* values were presented in Table S9. Of the 361 comparisons, 79 had significant differences (*p* < 0.05/19 = 0.0026) after Bonferroni correction, which were identified between Guizhou Tujia and Xinjiang Kyrgyz at 12 loci, followed by Xinjiang Uyghur at 10 loci, Xinjiang Mogolian at eight loci, Tibet Tibetan and Xinjiang Kazakh at seven loci, Guangxi Zhuang, Sichuan Tibetan, and Sichuan Yi at six loci, Guizhou Sui at five loci, Guangxi Mulao at four loci, Xinjiang Xibe at three loci, Ningxia Hui at two loci, and Shaanxi Han, Guizhou Han, Guizhou Miao at only one loci. No significant differences were observed between Guizhou Tujia and Xinjiang Han, Southern Han, Sichuan Han, and Guizhou Gelao. Significant differences were observed at DXS10159 locus of Guizhou Tujia and 19 reference populations, while no differences were found at DXS10074, DXS10134, and DXS10164 loci.

Pairwise Nei's genetic distances among 20 populations were estimated and listed in Table S10. The minimum genetic distance was found between Guizhou Tujia and Guizhou Gelao (0.0052), while Guizhou Tujia had the largest genetic distance with Xinjiang Mogolian (0.0891).

Then, phylogenetic relationships between Guizhou Tujia and other reference populations were explored using N‐J tree and MDS plot. As shown on the N‐J tree (Figure 1), three main branches were observed. The Mogolian‐speaking formed a single branch; Turkic‐speaking populations were clustered together in another branch, and the remaining (Sinitic, Hmong‐Mien, Tai‐Kadai, Tibeto‐Burman, Tungusic‐speaking) populations were gathered into the third cluster. Among the remaining five language speaking populations in the third branch, most people were also gotten together first adhering to their language family classification. Guizhou Tujia first combined with Guizhou Han and then grouped with Guizhou Miao and Gelao populations.

**FIGURE 1:** A neighbor‐joining tree based on the Nei's genetic distance among 20 Chinese population

The MDS (Figure 2) showed that Xinjiang Mogolian was located in the third quadrant and distant from the other 19 populations; the Tibeto‐Burman (except Guizhou Tujia) and Tungusic‐speaking populations were located in the first quadrant; three Turkic‐speaking populations were located in the second quadrant; Shaanxi Han, a Sinitic‐speaking population was located in the third quadrant but close to the populations in the fourth quadrant; and five Sinitic, four Tai‐Kadai, one Tibeto‐Burman, and one Hmong‐Mien speaking populations were located in the fourth quadrant. Guizhou Tujia, as one Tibeto‐Burman‐speaking population, was located in the fourth quadrant.

**FIGURE 2:** The multidimensional scaling (MDS) plot among 20 Chinese populations grouped into seven languages

Finally, PCA was also constructed with the exception of Xinjiang Mogolian populations, which can be prominently separated from others in the N‐J tree and MDS. As shown in Figure 3, 83.52% of total genetic variations were extracted from the first three principal components (PC1: 53.44%, PC2: 16.55%, PC3: 13.53%). PC1 separated Turkic language speaking people from others, and PC2 could differentiate six Sinitic language speaking populations and each language group clustered tightly. The third principal component showed a separation of Tai‐Kadai language speaking populations (except Guizhou Gelao) from the rest.

**FIGURE 3:** Principal component analysis (PCA) among 19 Chinese populations based on the PC1, PC2 and PC3

## 4 DISCUSSION

Herein, genotypes of 507 unrelated Tujia individuals (258 males and 249 females) from Guizhou were successfully obtained using AGCU X‐19 STRs PCR amplification kit. To explore the capacity of 19 X‐STRs in individual identification and forensic complex paternity testing, a series of forensic parameters were calculated, such as PDm, PDf, and four paternity exclusion chance (MEC_Krüger, MEC_Kishida, MEC_Desmarais, and MEC_Desmarais_Duos). MEC_Krüger (Krüger et al., 1968) indicated that all X‐chromosome markers of putative father can be identified and replaced by the putative grandmother in the deficiency paternity cases (unavailable putative father); MEC_Kishida (Kishida et al., 1997) and MEC_Desmarais (Desmarais et al., 1998) are appropriate for trios involving a female child. MEC_Desmarais_Duos (Desmarais et al., 1998) is valid for mother‐son kinship and father/daughter tests based on the X‐chromosome markers. In the present study, the combined PDm, PDf, and four paternity exclusion chances were all higher than 0.99999. Our findings indicate that 19 X‐STR loci have great information and polymorphism in Guizhou Tujia populations and the AGCU X‐19 STR kit can efficiently supplement the analyzes of other genetic markers (such as STRs, Y‐STRs, etc) in forensic and kinship analyses, especially in, cases involving females, such as mixed stains, deficiency paternity cases, and paternity cases involving blood‐relatives.

Genetic linkage is the tendency of two or more genetic markers of the same chromosome to remain together in the process of inheritance (Tillmar et al., 2017). X‐STR loci are all located on the X‐chromosome, it is necessary to consider the genetic linkage between any two loci when multiple X‐STRs were used in forensic cases (Tillmar et al., 2017). Linkage disequilibrium (LD) test, is a classical statistical method aiming to determine whether there is a genetic linkage state between different loci through analyzing non‐random association of alleles at different loci in a population (Tillmar et al., 2017). Which depends not only on physical/genetic distance but also on the factors affecting the population genetic structure, such as selection of marriage, random genetic drift, founder effect, population mixing or stratification, etc (Chakravarti, 1999). In our study, LD was analyzed both in males and females. There are five pairs (DXS10101‐DXS10075, DXS10103‐DXS10101, DXS10159‐DXS10162, DXS10162‐DXS10164, and DXS10162‐DXS7423) among 171 pairs of loci showed genetic linkage using LD test. Of the five pairs, three pairs (DXS10103‐DXS10101, DXS10159‐DXS10162, and DXS10162‐DXS10164) fell in the recognized linkage groups, while another two were between interlinkage groups. Tujia is a relatively isolated minority group due to the inconvenience of transportation in Guizhou province, so we speculate that the robust genetic linkage between two pairwise loci may attribute to the change of population genetic structure resulting from mating selection and genetic drift. According to the previous studies (Edelmann et al., 2002, 2010; Hering et al., 2006; Hundertmark et al., 2008; Samejima et al., 2011; Sufian et al., 2017; Szibor et al., 2005), 19 X‐STRs can be divided into seven linkage groups (LG). DNA Commission of the International Society for Forensic Genetics (ISFG) (Tillmar et al., 2017) recommends that haplotype frequencies of each linkage group should be adopted to calculate forensic parameters, which can obtain more reliable evidence in actual applications. The results show that each LGs is of high haplotype diversity genetic marker, and high discriminating efficiency can be provided when the seven LGs are jointly used in our studied population. Which further demonstrate that this kit can be used in actual complex parentage cases, including grandmother‐granddaughter duos, father‐daughter duos, mother‐son duos, half or full sibling duos involving two females, incest cases and so on.

Guizhou, a province inhabited by 56 ethnic groups officially recognized by Chinese government, has been a hot province in forensic genetics, anthropologists and ethnographers (Chen, He, Zou, Wang, Jia, et al., 2018; Chen, He, Zou, Wang, Luo, et al., 2018; Chen, He, Zou, Zhang, et al., 2018; Guo et al., 2019; Han et al., 2019; Le et al., 2019; Luo et al., 2019; Zhang et al., 2019). The population structures of Guizhou populations in different ethnic has been reported, particularly in Gelao (Chen, Han, et al., 2018; Chen, He, Zou, Wang, Jia, et al., 2018; Chen, He, Zou, Wang, Luo, et al., 2018), Han (Chen, He, Zou, Wang, Jia, et al., 2018), Miao (Chen et al., 2019; Han et al., 2019; Le et al., 2019; Zhang et al., 2019), and Bouyei (Luo et al., 2019; L. Zhang, 2015), but Tujia is unclear. In present study, we used various analytical methods (Fst, Nei's genetic distance, N‐J tree, MDS, and PCA) constructed population structure of Guizhou Tujia with diverse ethnic groups from seven major language families (Sinitic: Han, Hui; Tai‐Kadai: Gelao, Zhuang, Sui, Mulao; Tibeto‐Burman: Tibetan, Yi; Hmong‐Mien: Miao; Turkic: Uyghur, Kyrgyz, Kazakh; Mogolian: Mogolian; Tungusic: Xibe) in China. The overall consensus showed the characteristics of typical ethno‐linguistic and geographical clustering. For our studied people, Guizhou Tujia was relatively close to other indigenous populations living in Guizhou and surrounding provinces. Additionally, people who shared the same language have the intimate relationship except the Tibeto‐Burman language speaking populations.

The same and similar geographic and ethnolinguistic cluster characteristics observed in our study are also be reported using other genetic markers such as autosomal STRs and Y‐STRs In our previous phylogenetic relationship analysis using 15 autosomal STR loci among 27 Chinese ethnic groups based on the same statistical methods as our study (Gao et al., 2019), Guizhou Tujia was also close to the Sinitic language speaking populations and other ethnic groups living in Guizhou province, whereas far distant from the Tibeto‐Burman language speaking populations and the geographically distant populations. For the Y‐STR loci, although there is no population data of Guizhou Tujia reported up to date, by glancing over the other population studies based on different Y‐STR loci sets (Chen, Han, et al., 2018; Chen et al., 2019; Guan et al., 2020; Song et al., 2020; Tao et al., 2019), obvious consistence with the results of this study can easily be observed. For instance, Guizhou Gelao was close to geographically approximate Han populations, meanwhile both Tibetan and Mongolian ethnics assemble along their ethnolinguistic origin, respectively, but separated from other Chinese groups according to a study via 23 Y‐STR loci (Chen, Han, et al., 2018). Totally, our findings based on the 19 X‐STRs demonstrate that Guizhou Tujia are genetically similar with geographically close populations and other linguistically close populations, which is accordance with the autosomal STR and Y‐STR consequences of geography and language classification.

As commonly used genetic markers in forensic medicine, these three genetic markers showed a mixed clustering model: the Han populations from different administrative regions held together with geographical clustering of the Tujia and local Han populations in Guizhou. We speculated that they mainly experienced a long history of living together and inter‐mating in the Guizhou province. In addition, Guizhou Gelao is an indigenous ethnic minority in Guizhou province, which is geographically adjacent to the Guizhou Tujia. To further understand the migration and origin of the Tujia populations, and explore the elaborate genetic structure and subpopulation genetic structure in China, additional studies based on other genetic markers (SNP, Y‐STR, and mtDNA) in Guizhou and other provinces are needed.

## 5 CONCLUSION

In this study, we first analyzed the genetic polymorphisms of the Guizhou Tujia population based on AGCU X‐19 PCR kit. All loci in this population can be used to establish a reliable and informative database of X chromosome markers for human identification and paternity testing, especially in complex biological relations. Additionally, population comparisons indicate that Guizhou Tujia has genetic homogeneity with populations who reside in geographically adjacent regions and share the same language. Besides, Guizhou Tujia as a Tibeto‐Burman‐speaking population has an intimate relationship with geographically close Guizhou Gelao and the Han populations. Additional studies with other provinces and genetic markers of Tujia populations are needed for further understanding of the genetic structure of the Tujia populations.

## CONFLICT OF INTEREST

No potential conflict of interest was reported by the authors.

## AUTHOR CONTRIBUTIONS

PYC and LMY conceived the idea for the study. LL, HYG, LLY, HZ, and FL performed or supervised laboratory work. LL, LSZ, and LLY analyzed the data. PYC, LL, JY, and MLY wrote and edited the manuscript.

## Supporting information

Fig S1

Table S1‐S10
